RETRACTED

# Thermodynamic and kinetic insights into azo dyes photocatalytic degradation on biogenically synthesized ZnO nanoparticles and their antibacterial potential

**DOI:** 10.1016/j.heliyon.2024.e40679

**Published:** 2024-11-26

**Authors:** Abu Bakar Siddique, Muhammad A. Shaheen, Azhar Abbas, Yasir Zaman, Mohammed A. Bratty, Asim Najmi, Ali Hanbashi, Muhammad Mustaqeem, Hassan A. Alhazmi, Zia ur Rehman, Khalid Zoghebi, Hatem M.A. Amin

**Affiliations:** a Institute of Chemistry, University of Sargodha, Sargodha, 40100, Pakistan; b Department of Chemistry, Government Ambala Muslim College, Sargodha, 40100, Pakistan; c Department of Chemistry, Superior University, Sargodha Campus, Sargodha, 40100, Pakistan; d Department of Physics, University of Sargodha, Sargodha, 40100, Pakistan; e Department of Pharmaceutical Chemistry and Pharmacognosy, College of Pharmacy, Jazan University, Jazan, 82912, Saudi Arabia; f Department of Pharmacology, College of Pharmacy, Jazan University, Jazan, 82912, Saudi Arabia; g Health Research Center, Jazan University, Jazan, 82912, Saudi Arabia; h Chemistry Department, Faculty of Science, Cairo University, Giza, 12613, Egypt

**Keywords:** Zinc oxide NPs, Discoloration of MB and MO dyes, Carissa macrocarpa fruit extract, Radical scavengers, Photocatalyst

## Abstract

The extensive use of azo dyes in textile and pharmaceutical industries pose significant environmental and health risks. This problem requires to be tackled forthwith through a cheap, environmentally friendly and viable approach to mitigate water pollution. In this context, the green synthesis method was used for synthesis of ZnO NPs. These biogenic ZnO NPs were characterized by UV–Vis and Fourier transform infrared spectroscopy (FTIR), powder X-ray diffraction (PXRD), high-resolution transmission electron microscopy (HR-TEM) coupled with energy-dispersive X-ray (EDX), dynamic light scattering (DLS) and Zeta potential (ZP) analysis. The characteristic bandgap energy (3.02 eV), crystallite size (18.6 nm), particle size (84 nm), hydrodynamic diameter (101 nm) and ZP (−31.5 mV) all indicated the successful synthesis of the stabilized NPs, which have an absorption edge at 373 nm. Based on the responsive energy band gap to visible light, these NPs demonstrated promising photocatalytic activity for the degradation of toxic dyes with efficiencies of 82.2 and 87.5 % for of methylene blue (MB) and methyl orange (MO), respectively, in only 2 h of sunlight exposure. To evaluate the reaction kinetics and thermodynamic parameters including the activation energy and rate constant, the degradation process was conducted at various temperatures. The effect of temperature showed the highest rate constant values of 0.022 and 0.025 min^−1^ at 90 °C, and activation energies of 4.1 and 3.8 kJ mol^−1^ for MO and MB, respectively. A possible degradation mechanism was proposed based on results of the radical scavenging experiments. The photocatalyst showed recyclability for five consecutive cycles with a simple regeneration. CMFE@ZnO NPs have also exhibited great antibacterial potential by inhibiting the growth of Gram-positive (*S. aureus* (13 mm) and *B. subtilis* (14 mm)) and Gram-negative (*E. coli* (17 mm) and *P. multosida* (15 mm)) bacterial strains. As a result, these CMFE@NPs may have great commercial importance in reducing the concentration of azo dyes and drug-resistant bacteria in textile and pharmaceutical industry effluents.

RETRACTED

## Highlights

• Biosynthesis of *Carissa macrocarpa* fruit extract-mediated Zinc Oxide NPs (CMFE@ZnO NPs).
• Characterization of crystal parameters, colloidal stability and surface functionalization of ZnO NPs.
• Highly efficient photocatalyst for sunlight-driven degradation of azo dyes.
• Determination of kinetic and thermodynamic parameters of degradation.
• CMFE@ZnO NPs were more noxious to gram-negative bacterial strains.

## 1 Introduction

Azo dyes present in the effluents of textile, leather, and paper industries are one of the major pollutants that can have several detrimental effects on living organisms [1]. The toxicity of these dyes can affect the growth, reproduction, and survival of aquatic organisms such as fish, invertebrates, and algae [2]. Moreover, bioaccumulation of these dyes in tissues of aquatic organisms may disrupt the balance of whole ecosystem. The azo dyes can also pose a serious threat to health of human beings by causing skin irritation, allergic reactions, and potential carcinogenic effects [3]. Therefore, development of cheap, feasible and ecofriendly methods of wastewater treatment to mitigate the concentration of azo dyes in water effluents needs urgent attention.

Various technologies such as filtration, adsorption, reverse osmosis, and chromatography have been employed previously but degradation of azo dyes on photo-responsive nano catalysts under sunlight is considered to be a viable approach [4,5]. This method is ecofriendly, cheap, robust, and free of any hazardous chemicals to degrade dyes. Little or no energy and external chemical additions are required to treat wastewater.

Organic pollutants (azo dyes) are vulnerable to oxidation resulting in the decomposition of molecules, but molecular oxygen cannot directly oxidize many pollutants due to spin forbidden reactions, therefore activation of O_2_ to the more reactive species, called reactive oxygen species (ROS) is an interesting approach for pollutant remediation [6,7]. In this context, nanomaterials are important materials that can absorb the sunlight to excite valence electrons from valence band (VB) to conduction band (CB) and these segregated electron-hole pairs cause the redox reactions to generate ROS and degrade the azo dyes [8,9]. Various nanomaterials, such as TiO_2_ NPs [10,11], AgNPs [12,13], AuNPs [14] and heterostructures [15] like α-Fe_2_O_3_/g-C_3_N_4_/SiO_2_ [16] are being investigated nowadays but due to high cost of these materials, cost-effective ZnO NPs have emerged as an efficient alternative [17]. ZnO NPs are effective photocatalyst to degrade organic pollutants under sunlight due to their wide sunlight response, having energy bandgap in the range of 3.3 eV, high surface area and stable nature in form of colloidal solutions [18,19]. These NPs can easily generate ROS in aqueous media by absorption of light to excite electrons from the VB to CB. The ROS can degrade azo dyes and other pollutants by redox reactions and can ultimately mitigate the concentration of organic pollutants in the effluents of industries [20].

RETRACTED

Various approaches can be used to synthesize ZnO NPs such as hydrothermal, sol-gel, chemical precipitation, however the high cost and hazardous nature of reducing agents and energy consumptions are main limiting factors to use these techniques [21]. An alternative, non-toxic, cheap and viable method to synthesize ZnO NPs is the green approach using phytochemicals enriched extract as reducing and capping agent [22,23]. The greenly synthesized NPs are reported to have well defined morphology, monodisperse, highly stable and also biologically active to inhibit the growth of microbes. Various plant extracts enriched with phytochemicals especially phenolics and flavonoids have been utilized in past [24]. Ghaffar et al., reported the synthesis of ZnO NPs using olive fruit aqueous extract as effective photocatalyst to degrade different azo dyes in 3 h exposure to sunlight and biological applications [25], however higher exposure time can be further reduced by functionalizing the surface of NPs with various phytochemical enriched plant extracts. Therefore, quest for new plant extracts to synthesize NPs having desired properties is still an emerging field.

*Carissa macrocarpa (C. macrocarpa)*, commonly known as Natal plum is a tropical fruit-bearing plant native to South Africa. It is also widely found in the Asian region due to the use of its fruit in functional foods, dietary supplements, and natural health products [26,27]. The fruit of this plant is enriched in vitamins, fibers and phytochemicals, such as flavonoids, tannins, and phenolic compounds, which contribute to its antioxidant properties and potential health benefits. These valuable components are also found in the aqueous extract of this fruit as reported in the literature [28]. Hence, the aqueous extract can be used to reduce the salt ions to NPs and stabilized them by capping of phytochemicals on their surface.

RETRACTED

In addition to the photocatalytic applications, ZnO NPs are also reported to be good bactericidal agents, and their potential can be enhanced by the synergistic effect of phytochemicals coating and large surface area of NPs [29,30]. The NPs can inhibit the growth of bacteria by multiple routes, either by crossing the bacterial membranes due to their small size and interaction with DNA and growth proteins that results in the cell lysis, or by the generation of ROS on exposure to moisture and sunlight. These ROS can easily induce oxidative stress in bacterial cells, leading to damage to proteins, lipids, and DNA, ultimately causing bacterial cell death. These properties have led to the exploration of ZnO NPs in various applications, such as antibacterial coatings, wound dressings, and water disinfection systems [31,32].

Inspired from the promising physicochemical and biological properties of biogenic ZnO NPs and since no previous studies have reported on synthesis of ZnO NPs using phytochemical enriched *Carissa macrocarpa* fruit extract (CMFE), the current research was focused on the green synthesis of ZnO NPs using CMFE. The as-synthesized ZnO NPs were characterized by modern analytical techniques such as XRD, UV–Vis., FTIR, HR-TEM, EDX, DLS, and ZP analysis. Upon successful characterization, the NPs were employed as an effective photocatalyst to decompose MB and MO dyes under sunlight radiation. The reusability studies were carried out to estimate the potential of NPs for repeated usage after efficient regeneration step. Importantly, the kinetics and thermodynamic parameters of degradation were assessed. Furthermore, radical scavenging experiments were carried out to elucidate the underlying degradation mechanism. The antibacterial efficacy of as-synthesized ZnO NPs has also been evaluated by the disc diffusion assay against different bacterial strains.

## 2 Experimental

### 2.1 Materials and methods

All chemicals, including zinc nitrate (Zn(NO_3_)_2_.6H_2_O), sodium hydroxide (NaOH), hydrochloric acid (HCl) and chromic acid (H_2_Cr_2_O_7_) were purchased from Merck, Germany. Deionized water was used for preparations of all solutions.

The Shimadzu FTIR-8400S spectrophotometer (Japan) and Shimadzu UV-1800 spectrophotometer (Japan) were used to record the FTIR and UV–Vis spectra of samples in the range of 4000–400 cm^−1^ and 200–800 nm, respectively. Zetasizer Nano ZS (Malvern Panalytical) was used for DLS and ZP measurements. X-ray diffraction pattern was recorded on the diffractometer JDX-3532, JEOL, Japan, with Cu-Kα lines (wavelength of 1.5418 Å) over a 2θ range of 10–80°. TEM images were obtained using HR-TEM (JEM-ARM2000F, JEOL, Japan) for morphological analysis of samples.

RETRACTED

### 2.2 Preparation of CMFE

*C. macrocarpa* fruit extract (CMFE) was synthesized following the previously reported literature [33,34]. In summary, *C. macrocarpa* fruits were washed, shredded and dried in shade for three weeks and grinded to fine powder. The powder (20 g) was homogenized in 0.5 L distilled water and subjected to reflux for 2 h at 100 °C. Subsequently, phytochemicals enriched aqueous phase was separated by filtration and dried to powder by evaporation at 60 °C for 24 h. This powder was used for further analysis and synthesis of NPs.

### 2.3 Phytochemical screening of CMFE

Qualitative phytochemical screening of the extract was performed using standard tests of phenolics, carbohydrates, tannins, flavonoids, terpenoids, saponins, terpenoids, anthraquinone and alkaloids. Prominent color changes according to the reported methods for screening affirmed the presence of specific phytochemicals in the samples.

Lead acetate Test was used to check the presence of phenolic content [35]. The extract (2 mL) was mixed with the lead acetate solution (10 %, 1 mL) and the appearance of white color precipitates indicated the presence of phenols.

For confirmation of carbohydrates, Molisch Test was performed [36]. The freshly prepared extract (2 mL) was mixed with 2 mL of Molisch's reagent. After proper shaking, 2 mL of concentrated sulfuric acid was added alongside the wall of test tube. Appearance of violet ring at the interface confirmed the presence of carbohydrates.

Tannins were identified by Braymer's Reagent Test [37]. The mixing of aqueous FeCl_3_ solution (2 %, 2 mL) in extract (1 mL) showed the appearance of greenish black color, indicated the presence of tannins.

Flavonoids were tested by Shinoda Test [38]. The appearance of pink, scarlet color after addition of magnesium ribbon along with the concentrated HCl dropwise (3 mL) in the extract (2 mL) indicated the presence of flavonoids.

Terpenoids were tested by Salkowski Test [38]. The extract (1 mL) was mixed with the 2 mL of chloroform followed by the addition of 2 mL of H_2_SO_4_, resulting in the appearance of reddish-brown color on gentle shaking. Reddish brown color showed the presence of steroidal ring in the extract.

The presence of saponins was confirmed by the Foam Test [39]. The extract (3 mL) was diluted with distilled water (5 mL) followed by vigorous shaking resulted in the formation of stable foam, proved the presence of saponins.

RETRACTED

Borntrager Test was used to check the presence of anthraquinones in the extract [40]. The extract (5 mL) was boiled in dilute sulfuric acid and filtered. Filtrate was extracted in chloroform and few drops of strong ammonia solution were added in it. After few min, the appearance of pink color indicated the presence of anthraquinones in extract.

Draggendorff Test was used for indication of alkaloids [38]. The change of extract color from pink to brown by adding a few drops of Draggendorff reagent to the extract (2 mL) indicated the presence of alkaloids.

### 2.4 Synthesis procedure of CMFE@ZnO NPs

For the synthesis of CMFE@ZnO NPs, separate solutions of Zn(NO_3_)_2_.6H_2_O (50 mM, 50 mL) and CFME (30 mg/15 mL, 15 mL) were prepared in deionized water. Then, the aqueous extract and salt solution were mixed at constant stirring rate of 200 rpm and a pH 9 was maintained by addition of 0.1 M solution of NaOH. The resulting mixture was heated at 80 °C for 40 min under constant stirring at 200 rpm. The formation of white color precipitates indicated the synthesis of ZnO NPs. The ZnO NPs were separated from mixture by centrifugation at 8000 rpm for 30 min and rinsed thrice with deionized water. Afterwards, CMFE@ZnO NPs were oven dried at 75 °C for 4 h, followed by calcination at 350 °C for 2 h in muffle furnace. The UV–Vis spectra of these NPs sonicated in distilled water showed the characteristic peak of ZnO NPs at 373 nm.

### 2.5 Photocatalytic activity evaluation of CMFE@ZnO NPs

Photocatalytic potential of greenly synthesized CMFE@ZnO NPs was evaluated to degrade MB and MO dyes under sunlight irradiation following the reported method [41]. In brief, the adsorption-desorption equilibrium was initially developed on the surface of catalyst by stirring the CMFE@ZnO NPs (20 mg) with dye solution (20 mL, 10 ppm) for 30 min at 200 rpm. Afterwards, this combination was exposed to sunlight for 120 min, which caused the color to continuously fade. The % degradation of dye was calculated by measuring the absorbance of solution in 15 min interval at ambient temperature (25 ± 2 °C), using Equation (1).

(1) $$\%\;\text{dye}\;\text{degradation}=\frac{C_{0}-C_{f}}{C_{0}}\times 100=\frac{A_{0}-A_{f}}{A_{0}}\times 100$$

where, *C*_*0*_ is the initial concentration and *C*_*f*_ is the concentration of dye after time *t*. The absorbance spectra of MB and MO solutions were recorded at the *λ*_max_ of 668 nm and 465 nm, respectively.

### 2.6 Effect of reaction parameters on photodegradation rate

Photodegradation of organic pollutants is highly dependent on catalyst dose, pH and water composition. In order to evaluate the effect of these parameters and optimize the reaction conditions, batch experiments of photodegradation of MB and MO dyes were carried out in the pH range of 3–11, catalyst dosage of 1–20 mg and in various water composition samples (spiked distilled water (DW), tap water (TW), and river water (RW)) following the same procedure as described above.

RETRACTED

### 2.7 Reusability study of the photocatalyst

Reusability experiments of the CMFE@ZnO NPs were conducted for five consecutive cycles for the photodegradation of dyes in order to verify the catalyst's recyclability. The catalyst was recovered and activated following the reported procedure after each cycle [41]. In short, after each degradation experiment, the mixture was centrifuged and filtered to separate the catalyst. The catalyst was then dried at 80 °C for 4 h and was reused for subsequent experiments.

### 2.8 Antibacterial efficacy of CMFE@ZnO NPs

The bactericidal activity of CMFE and CMFE@ZnO NPs was investigated using the disc diffusion method [42]. In summary, agar solution (3 g/100 mL H_2_O) was used to develop four bacterial strains: 2 gram-negative strains (*Escherichia coli* and *Pasturella multosida*) and 2 gram-positive strains (*Staphylococcus aureus* and *Bacillus subtilis*). The colonies were cultured for 24 h at 4 °C, followed by the adjusting the mixture's turbidity at 108 CFU using 0.9 % saline. After autoclaving the plates for an hour at 120 °C, the pre-grown bacterial colonies were seeded into the petri dishes filled with agar. 1 mL of aqueous CMFE (2 mg/5 mL) solution and CMFE@ZnO NPs (2 mg/5 mL) was placed on separate sterilized paper discs and these discs were arranged on petri dishes. A paper disc loaded with distilled water was used as negative standard. To assess the bacterial inhibition, these petri dishes were incubated for the following 24 h at 37 °C. On next day, each disc's zone of inhibition was measured in millimeters (mm).

### 2.9 Statistical analysis

ANOVA was used to assess the statistical significance of each experiment by repeating each experiment thrice. The findings were presented with a statistical significance threshold of p < 0.05, expressed as mean ± standard deviation.

## 3 Results and discussion

### 3.1 Phytochemical screening of CMFE

The phytochemical screening of the CMFE was carried out to check the presence of phenolic content, flavonoids, terpenoids, sugars, alkaloids, anthraquinones, etc. These phytochemicals play an important role in reducing the metal ions and stabilizing the formed NPs by capping their surface. The results of screening tests revealed the phytochemical-enriched nature of CMFE (Table 1). The presence of these bioactive species in the extract also imparts the biological importance, i.e., antimicrobial properties to the synthesized NPs.

RETRACTED

**Table 1:** Phytochemical screening results for the CMFE extract.

**Metabolite**	**Test**	**Observation**	**Result**
**Phenols**	Lead acetate test	white precipitates	Positive
**Carbohydrates**	Molisch test	violet ring	Positive
**Tannins**	Braymer's reagent test	greenish black color	Positive
**Flavonoids**	Shinoda test	pink scarlet color	Positive
**Terpenoids**	Salkowski test	pink scarlet color	Positive
**Saponins**	Foam test	stable foam	Positive
**Anthraquinones**	Borntrager test	pink color	Positive
**Alkaloids**	Draggendorff test	brown color	Positive

#### 3.1.1 UV–Vis and FTIR analyses

The UV–Vis spectrum of the CMFE@ZnO NPs was recorded in the range of 200–800 nm after sonicating the solid ZnO NPs in water for 10 min. The UV–Vis spectra of finely dispersed CMFE@ZnO NPs and bare CMFE are shown in Fig. 1a.

**Fig. 1:** **(a)** UV–Vis spectra of neat CMFE and CMFE@ZnO NPs, **(b)** Tauc's plot of CMFE@ZnO NPs.

The UV–Vis absorbance spectrum showed the characteristic peak of ZnO NPs at 373 nm in the aqueous solution of zinc nitrate and CMFE, while no specific prominent peak was noticed in the spectrum of neat CMFE solution. Moreover, no characteristic peak of ZnO NPs around 370 nm was observed in the control solution of zinc nitrate without CMFE after 40 min of mixing, as shown in Fig. S1, suggesting the essential role of the extract in the formation of such NPs. The characteristic peak of ZnO NPs peak is due to the surface plasmon resonance (SPR) phenomenon at these plasmonic ZnO NPs. This peak is observed due to the collective oscillations of electrons in the conduction band on interaction with electromagnetic radiations [43]. It was anticipated that CMFE@ZnO NPs were formed by three step reaction via a green synthesis approach as previously reported in the literature [44]. In the 1^st^ step, the complexation of zinc (II) ions occurs with the phytochemicals of the CMFE. In the 2^nd^ step, the thermal degradation of zinc complex occurs at high temperature, resulting in the formation of ZnO NPs. In the 3^rd^ step, these ZnO NPs were functionalized with the functional groups of various phytochemicals, resulting in the synthesis of CMFE@ZnO NPs [44]. The brief mechanism of formation of CMFE@ZnO NPs is depicted in Fig. S2.

Furthermore, the Tauc's plot was established from the absorbance data to calculate the bandgap energy utilizing Equation (2).

(2) $$\alpha hv=B{\left(hv-E_{g}\right)}^{\gamma }$$

Where, *α, hν, E*_*g*_ and *B* represent the absorption coefficient, photon energy, optical bandgap energy and a constant. The value of α can be determined using Equation (3).

(3) $$\alpha =\frac{2.303\;A}{t}$$

Where, *A* is the absorbance and *t* is the path thickness. γ in Equation (2) is the Tauc's exponent. Its value is 0.5 for direct energy bandgap. Accordingly, from the plot of *(αhυ)*^*2*^ against *hυ*, a direct bandgap energy (*E*_*g*_) value of 3.02 eV was obtained, as shown in Fig. 1b. The bandgap energy value (3.02 eV) indicated the absorbance of visible light for the excitation of electrons from the valence band (VB) to the conduction band (CB) and the generation of charge carriers in the lattice.

RETRACTED

FTIR spectra of CMFE and CMFE@ZnO NPs were recorded to determine the major functional groups on the surface of CMFE@ZnO NPs and in the neat extract, as shown in Fig. 2. The spectrum of CMFE showed the presence of many functional groups’ peaks, i.e., aromatic ring (C=C), carbonyl group (C=O), atmospheric CO_2_, alkyl groups (C-H), and hydroxyl group (O-H) at 1450, 1690, 2310, 2940 and 3250-3600 cm^−1^, respectively [42]. The presence of peaks of many functional groups on the surface of CMFE@ZnO NPs indicates the successful capping of the surface of NPs. In addition to the above-mentioned peaks, a new peak around 500 cm^−1^ assigned to Zn-O was also observed in the spectrum of CMFE@ZnO NPs.

**Fig. 2:** FTIR spectra of CMFE and CMFE@ZnO NPs.

#### 3.1.2 XRD, HR-TEM and EDX characterization

As can be seen in Fig. 3a, the PXRD spectrum of CMFE@ZnO NPs was obtained in the 2θ range of 10–80°. According to JCPDS File No. 36–1451, Bragg's reflections observed at 2θ values of 31.7°, 34.3°, 36.2°, 47.4°, 56.5°, 62.8°, and 67.8° were assigned to crystal planes (100), (002), (101), (102), (110), (103), and (112), respectively. These strong Bragg's reflections confirmed the hexagonal crystal structure of CMFE@ZnO NPs with space group *P*6_3_*mc* (186). The Debye-Scherrer relation (Equation (4)), the dislocation density (δ) formula (Equation (5)), the micro strain (ε) formula (Equation (6)) and the degree of crystallinity (Equation (7)) were used to compute the crystal parameters, which include crystallite size, dislocation density, micro strain and degree of crystallinity, respectively. The values of these parameters are depicted in Table 2.

(4) $$D=\frac{K\lambda }{\beta \;\cos\;\theta }$$

(5) $$\delta =\frac{1}{D^{2}}$$

(6) $$\varepsilon =\frac{\beta }{4\;\tan\;\theta }$$

(7) $$\text{Degree}\;\text{of}\;\text{crystallinity}=\frac{\text{Area}\;\text{of}\;\text{crystalline}\;\text{peaks}}{\text{Area}\;\text{of}\;\text{all}\;\text{peaks}}\times 100$$

Where *D*, *λ*, *θ*, *β* and *K* represent the crystalline size, X-ray wavelength (Cu κα = 0.154 nm), diffraction angle, FWHM, and shape factor or Scherrer constant (typically 0.9), respectively.

RETRACTED

**Fig. 3:** (a) PXRD spectrum of CMFE@ZnO NPs; (b) EDX analysis of CMFE@ZnO NPs; (c) HR-TEM image of CMFE@ZnO NPs and (d) Histogram of particle size distribution of CMFE@ZnO NPs.

**Table 2:** Crystal parameters of CMFE@ZnO NPs.

**Sample**	**Average crystallite size *D* (nm)**	**Dislocation density δ×10**^**−3**^**(nm**^**−**^**^2^)**	**Micro strain** **ε×10**^**−3**^	**Degree of Crystallinity (%)**
**CMFE@ZnO NPs**	18.6	2.9	0.7	94.1

Furthermore, the morphological and elemental composition analysis of the CMFE@ZnO NPs were carried out using HR-TEM and EDX, respectively. The HR-TEM image of the CMFE@ZnO NPs was captured to analyze the shape and particle size of the particles, as shown in Fig. 3c. The TEM image revealed the appearance of monodispersed NPs with irregular shape, but with dominating spherical particles. TEM images were analyzed to calculate the particle size distribution, and the average particle size as depicted in the histogram in Fig. 3d. The average particle size of CMFE@ZnO NPs was found to be 83.6 ± 12.9 nm. In addition, the EDX spectrum (Fig. 3b) of CMFE@ZnO NPs showed the evident main peaks of Zn at 1.01 and 8.63 keV and oxygen at 0.52 KeV. In addition to these peaks, peaks of different elements including C, Na, Al, Si, Cl, and K were also observed due to the various bioactive compounds in the capping agent on the surface of CMFE@ZnO NPs. These additional peaks are generally observed in the greenly synthesized NPs [45]. Si and Al are from the sample holder.

#### 3.1.3 Hydrodynamic diameter and colloidal stability of CMFE@ZnO NPs

The hydrodynamic diameter and surface charge of CMFE@ZnO NPs were ascertained by dynamic light scattering (DLS) and Zeta potential (ZP) measurements, as illustrated in Fig. 4. As presented in Fig. 4a, the DLS measurement analysis revealed a narrow particle size distribution in the 70–130 nm range. The average hydrodynamic diameter was found to be 100.5 ± 18.4 nm. The particle size estimated by HR-TEM analysis was found to be comparatively smaller than the hydrodynamic diameter. The reason for this difference is the hydration of CMFE@ZnO NPs in the aqueous medium,where in the DLS measurement the particle size with the surrounding hydration shell is measured.

**Fig. 4:** (a) DLS analysis data and (b) Zeta potential analysis data of CMFE@ZnO NPs.

Based on ZP analysis, the average ZP value by surface charge determination was found to be −31.5 ± 3.1 mV, as illustrated in Fig. 4b. This value implies a negative charge on the particles’ surface, causing repulsion among them and hence promoting their colloidal stability in the liquid phase. Based on this relatively high ZP value, the suspensions are electrostatically stable and resistant to agglomeration in the aqueous media.

RETRACTED

### 3.2 Photocatalytic degradation of MB and MO at CMFE@ZnO NPs under sunlight

One feasible method to remediate azo dyes is their photocatalydtic degradation using visible light-responsive nanomaterials. These nanomaterials should have the bandgap energy between 1.63 and 3.26 eV to generate electron-hole pairs that produce radicals and reactive oxygen species (ROS), which subsequently photodegrade toxic azo dyes. The as-synthesized CMFE@ZnO NPs have the potential to photocatalytically degrade MB and MO dyes under direct solar radiation due to their suitable bandgap energy of 3.02 eV and their high surface area. To monitor the photocatalytic degradation, the UV–Vis spectra were measured after every 15 min for 120 min of sunlight exposure. Fig. 5a and b clearly illustrate the gradual decline in the absorption intensity of the distinctive peaks of azo dyes, namely 668 nm for MB and 465 nm for MO. The absorption almost vanishes after 180 min.

**Fig. 5:** Absorbance spectra of dyes solution at different times of sunlight exposure for (a) MB dye and (b) MO dye; (c) % degradation of dyes versus time. (d) pseudo-first order kinetics graphs of degradation of MB and MO dye at ambient temperature (25 ± 2 °C).

To evaluate the degradation percentage, dye degradation was calculated using Equation (1) for each time interval. As can be clearly seen in Fig. 5c, the degradation % of MB and MO dyes steadily increases with time, achieving 82.2 % and 87.5 %, respectively, after 120 min under sunlight. Furthermore, the kinetics of degradation were studied. Equation (9) was used to fit the degradation data to pseudo first-order kinetics to get a deeper understanding of the kinetics of degradation.

(9) $$\ln\frac{C}{C_{o}}=kt$$

The degradation data was well fitted into Equation (9) with *R*^*2*^ values of 0.981 and 0.982 for MB and MO dye, as shown in Fig. 5d. The slope of this plot gives the degradation rate constant (*k*) and values of 1.49 x 10^−2^ min^−1^ and 1.77 x 10^−2^ min^−1^ were obtained for MB and MO dye, respectively. To compare the performance of our photocatalyst with previously reported relevant photocatalysts, a summary of the percentage of dye degradation and rate constants is presented in Table 3. The comparison manifested better or at least comparable degradation percentages as well as rate constants for our catalyst compared to previous materials. Importantly, this photocatalyst outperforms other materials in that it needed only 120 min to achieve 88 and 82 % degradation under direct sunlight, which is much shorter time than many others (see Table 3). These results hint to the promising potential of the synthesized material as a photocatalyst.

RETRACTED

**Table 3:** Comparison of photocatalytic potential of CMFE@ZnO NPs with previously reported ZnO based materials for the degradation of MB and MO dye.

**Material**	**% Dye Degradation/rate constant k (min**^**−**^**^1^)**		**Conditions**	**Reference**
	**MB Dye**	**MO Dye**		
ZnO	84/0.035	88/0.012	150 min for MB & 60 min for MO under UV lamp	[46]
Fe-doped ZnO	–	82/0.025	90 min in sunlight	[47]
ZnO-GO	92.5/0.023	–	120 min under UV light irradiation	[48]
ZnO@OFE	75/0.008	87/0.013	180 min in sunlight	[25]
Carbon doped ZnO NPs	90.3/0.0207	–	300 min under a 500 W metal halide lamp with a 420 nm cut off filter	[49]
ZnO-rGO	88/---	–	260 min under UV-Lamp	[50]
CMFE@ ZnO NPs	82.2/0.015	87.5/0.018	120 min in sunlight	This work

#### 3.2.1 Effect of pH, catalyst dosage and water composition on photodegradation

It is well reported that the pH of the reaction media greatly affects the degradation efficiency by altering the surface charge of dyes and catalyst, formation of different ions in the medium and affecting the adsorption capacity of dyes on catalysts. From Fig. 6a, it can be seen that the % degradation of dyes was maximum around pH 7. Above pH 7, the % degradation decreased because in high alkaline media, the hydrolysis of ZnO NPs prevails, resulting in the lowering of the surface area of the catalyst as well as a decrease in the number of active sites. While below pH 7, the % degradation of cationic dye (MB) has continuously decreased because the adsorption capacity decreased with decreasing the negative charge density on CMFE@ZnO NPs. The adsorption capacity of MO (anionic dye) increases below pH 7, but the % degradation still decreases slowly. This can be explained on the fact that the predominant hydrogen ions present in the acidic media can easily scavenge hydroxyl radicals, which results in the lowering of % degradation.

**Fig. 6:** (a) Effect of pH, (b) catalyst dose and (c) water composition on % dye degradation of MB and MO dyes at ZnO NPs photocatalyst.

The effect of catalyst dosage revealed that the catalytic efficiency increases with the increase of the catalyst dosage due to an increase of active sites but then decreases for dosages beyond 10 mg, as can be seen in Fig. 6b. A decrease in % degradation was observed because at high catalyst dosage, the turbidity of media is increased, and light penetration is sufficiently decreased. High catalyst dose may also result in the higher agglomeration of NPs.

From Fig. 6c, the effect of water composition on photodegradation revealed that the maximum % degradation was observed in spiked DW as compared to TW and RW solutions due to the absence of interferences, like absence of interfering ions and other organic impurities as well as low turbidity of spiked DW.

RETRACTED

#### 3.2.2 Kinetics and thermodynamics of dye degradation

The catalytic reactions were subsequently carried out at various temperatures in the range of 30–90 °C (Fig. 7a and b) in order to gain a greater understanding of the reaction kinetics and thermodynamic properties, i.e., activation energy (*E*_*a*_), enthalpy change (*ΔH*), entropy change (*ΔS*), and Gibbs free energy change (*ΔG*). The values of various thermodynamic parameters were determined using Equations (10), (11), (12), (13), (14)). The values of the rate constant at various temperature was determined by plotting the ln*(A*_*t*_*/A*_*0*_*)* versus reaction time as shown in Fig. 7a and b. Afterwards, the *E*_*a*_ value was determined by plotting the ‘ln k’ vs ‘1/T’ as shown in Fig. 7c.

(10) $$\ln\left(A_{t}/A_{0}\right)=–kt$$

(11) $$\ln\;k=\ln\;A–E_{a}/RT$$

(12) $$\Delta H=E_{a}\;–\;RT$$

(13) $$\ln\left(k/T\right)=–\Delta H/\;RT+\Delta S/\;R+\ln\left(k_{B}/h\right)$$

(14) ΔG=ΔH–TΔS

Here*, k, t, R, T, K*_*B*_ and *h* represent the rate constant, time, ideal gas constant, temperature, Boltzmann constant and Planck's constant, respectively. The activation energy (*E*_*a*_), enthalpy change (*ΔH*), entropy change (*ΔS*), and Gibbs energy change (*ΔG*) values of MO and MB degradation are shown in Table 4, respectively. Positive values of *E*_*a*_ and ΔG for both dyes indicated the endothermic and non-spontaneous nature of the catalytic process, respectively. The value of *E*_*a*_ of about +4 kJ mol^−1^ obtained at this photocatalyst suggests that the catalyst lowered the activation barrier needed for the photodegradation to occur.

**Fig. 7:** Effect of temperature on reaction kinetics of **(a)** MB dye degradation and **(b)** MO dye degradation, **(c)** Arrhenius plot for the determination of *E*_*a*_ of degradation of dyes at ZnO NPs.

**Table 4:** Thermodynamic parameters for the degradation of MO and MB dyes on ZnO NPs.

**Dye**	***T* (K)**	***E***_***a***_**(kJ mol**^**−**^**^1^)**	***ΔH* (kJ mol**^**−**^**^1^)**	***ΔS* (J mo1**^**−**^**^1^** K^–1^**)**	***ΔG* (kJ mol**^**−**^**^1^)**
**MO**	303	4.1	1.5	−272.6	84.1
	323		1.41	−273.9	89.9
	343		1.24	−274.4	95.4
	363		1.08	−274.1	100.5
**MB**	303	3.8	1.28	−274.5	84.5
	323		1.11	−275.3	90.0
	343		0.94	−275.8	95.5
	363		0.78	−276.0	101.1

#### 3.2.3 Effect of radical scavengers and proposed mechanism

Organic pollutants are quickly degraded by reactive oxygen species (ROS), which include hydroxyl radicals (HO^•^), superoxide anion radicals (O_2_^−•^), hydrogen peroxide (H_2_O_2_), and holes (h^+^) [51]. In batchwise radical scavenging tests, the production and major contributing species involved in degradation were assessed. The analyses used four scavengers: p-benzoquinone (p-BQ) for O_2_^−•^, isopropanol (IPA) for HO^•^, disodium ethylenediamine acetate (Na_2_EDTA) for h^+^, and L-ascorbic acid (L-AA) for H_2_O_2_ [52]. In every run of the experiment, 20 mg of catalyst was added to a 10 ppm dye solution (20 mL), and 10 mL of a 0.2 mM solution of one radical scavenger was dissolved in it. The previously discussed method was used to monitor each dye's rate of degradation.

RETRACTED

By radical scavenging experiments, it was observed that the % dye degradation was decreased in the presence of all radical scavengers, which reflected that all the reactive species were produced in the solution under sunlight, as shown in Fig. 8. However, in the presence of IPA and Na_2_EDTA, minimal degradation of dyes was observed, which means that the OH^**•**^ and h^+^ were majorly involved in the degradation of dyes on the surface of the catalyst.

**Fig. 8:** Effect of radical scavengers on the degradation of MB and MO dyes.

For further insight of electron transfer and degradation mechanism, VB and CB edge potentials were calculated by Butler – Ginley equations (Equation (15), (16)) [53].

(15) $$E_{CB}=X-E_{C}-0.5E_{g}$$

(16) $$E_{VB}=E_{CB}+E_{g}$$

Here, *E*_*C*_*, E*_*g*_ and *X* represent the energy of free electrons (4.5 eV), bandgap energy (3.02 eV) measured by Tauc's plot and Mulliken's absolute electronegativity (5.71 for ZnO), respectively. The values of *E*_*CB*_ and *E*_*VB*_ were found to be −0.29 V and +2.72 V, respectively as shown in Scheme 1. These band edge positions showed that the generation of ^**•**^OH is most feasible due to oxidation potential of OH^−^/^**•**^OH is +2.4 V and E_VB_ is present at +2.72 V. This finding also supported the experimental results of radical scavenging experiments because minimum degradation of dyes was observed on scavenging of in ^**•**^OH in presence of IPA.

**Scheme 1:** Photocatalytic degradation mechanism at ZnO NPs showing the position of valence band and conduction band along with feasible electron transfer mechanism and redox reaction with dye.

By analyzing the effect of these radical scavengers in the degradation process, the degradation mechanism of azo dyes was proposed, as shown in Equations (17), (18), (19), (20), (21), (22), (23), (24), (25)). It was postulated that, the valence electrons of the catalyst are excited to conduction band in presence of sunlight radiations, resulting in the production of e^−^ and h^+^ pairs. The e^−^ are absorbed by the dissolved oxygen, and the h^+^ reacts with water to produce OH^**•**^ radicals. Several secondary radicals are produced in the mixture by secondary reactions and actively participate in the degradation phenomenon. involved in dye degradation.

(17) $$ZnO+hv\to ZnO\;\left(e^{-}\left(CB\right)+h^{+}\left(VB\right)\right)$$

(18) $$H_{2}O\;\left(ads\right)+h^{+}\;\left(VB\right)\to {OH}^{\cdot }\left(ads\right)+H^{+}\left(ads\right)$$

(19) $$O_{2}+e^{-}\left(CB\right)\to O_{2}^{-\cdot }\left(ads\right)$$

(20) $$O_{2}^{-\cdot }\left(ads\right)+H^{+}⇆{HOO}^{\cdot }\left(ads\right)$$

(21) $${HOO}^{.\;}\;\left(ads\right)\to H_{2}O_{2}\left(ads\right)+O_{2}$$

(22) $$H_{2}O_{2}\;\left(ads\right)\to 2{OH}^{\cdot }\;\left(ads\right)$$

(23) $$Dye+2{OH}^{\cdot }\to intermediates\to CO_{2}+H_{2}O$$

(24) $$Dye+h^{+}\left(VB\right)\to Oxidation\;products$$

(25) $$Dye+e^{-}\left(CB\right)\to Reduction\;products$$

RETRACTED

#### 3.2.4 Regeneration of the photocatalyst

Using the previously described method [54], the reusable nature of the photocatalyst was assessed for the degradation of azo dyes for five consecutive cycles. In summary, the catalyst, i.e., CMFE@ZnO NPs, was recovered by a simple regeneration step comprising centrifugation of the mixture for 30 min at 3000 rpm. The solid catalyst was reused after rinsing three times with distilled water and drying for 4 h at 80 °C. The regeneration study's results (Fig. 9a) demonstrated the catalyst's stability and capability for reuse with a minimal decay in performance. After multiple usages, mere 10 % decrease in activity proved the catalyst's effectiveness for repeated usage. After appropriate activation, it seems that the described catalyst can be utilized several times for wastewater treatment.

**Fig. 9:** (a) Reusability studies of CMFE@ZnO NPs for the degradation of MB and MO over 5 consecutive cycles. (b) Antibacterial activity results of CMFE, CMFE@ZnO NPs and negative control (water).

### 3.3 Antibacterial potential of CMFE@ZnO NPs

Using the disc diffusion test, the antibacterial efficacy of CMFE and CMFE@ZnO NPs was assessed against 2 g-positive strains (*S. aureus* and *B. subtilis*) and 2 g-negative strains (*E. coli* and *P. multosida*). Because CMFE contains a variety of phytochemicals, including phenolics, flavonoids, alkaloids, terpenoids, etc., it has been speculated that it has antibacterial potential [26]. Furthermore, the NPs can easily pass-through cell barriers and interact with growth proteins and genetic material, they can also stop the growth of some bacterial strains [51]. The synergistic impact of successfully encapsulating NPs with phytochemical species greatly enhances their antibacterial efficacy [55,56]. Thus, a comparison of CMFE and CMFE@ZnO NPs' antibacterial activities was conducted.

RETRACTED

The results of the zone of inhibitions showed that, in comparison to CMFE, the CMFE@ZnO NPs were more effective to inhibit the growth of the bacterial strains as shown in Fig. 9b. It's interesting to note that CMFE@ZnO NPs had shown more deterioration to gram-negative strains of bacteria. The exact mechanism of mode of action of ZnO NPs against bacterial cells is still undiscovered. However, different types of interactions of NPs with bacterial cells have been reported in literature, mainly the interactions of NPs with bacterial cell wall resulting in the more penetration of small size NPs, release of Zn^2+^ ions inside the cells, ROS generation at cell wall and inside the cell, interactions with proteins and nucleic acids and disruption of metabolic pathways [57,58]. The CMFE@ZnO NPs' remarkable activity against gram-negative bacteria was ascribed to the variations in the cell membranes of the bacterial strains. Gram-negative bacteria have very thin cell walls, which make it easier for tiny particles to pass through and prevent the cell from normal functioning [58,59]. There was a greater suppression of gram-negative bacterial strains as a result of the enhanced entry of CMFE@ZnO NPs within the cells and the combined action of NPs and capping agents to restrict the normal functioning of cell by irreversible attachment to proteins and nucleic acid as well as ROS generation inside the cell.

## 4 Conclusions

Herein, greenly synthesized CMFE@ZnO NPs is reported as an eco-friendly, cheap and feasible sunlight driven photocatalyst for the degradation of toxic azo dyes and as an antibacterial agent. Appropriate bandgap energy (3.02 eV), narrow particle size distribution (83.6 ± 12.9 nm), and high colloidal stability (zeta potential of −31.5 ± 3.1 mV) have solidified the basis for this material to be employed as a photocatalyst. The catalyst showed high photocatalytic activity by degrading methylene blue (82.2 %) and methyl orange (87.5 %) in just 2 h of exposure to direct sunlight following pseudo-1^st^ order kinetics. The rate constant (*k*) was found to be 1.49 x 10^−2^ min^−1^ and 1.77 x 10^−2^ min^−1^ for MB and MO dye, respectively, which is relatively high compared to that of previously reported relevant catalysts. Additionally, the photocatalyst demonstrated low activation energy (4.1 and 3.8 kJ mol^−1^) for the degradation of MB and MO dye, respectively. Furthermore, the radical scavenging experiments showed that the HO^**•**^ and h^+^ are major reactive oxygen species involved in the degradation of pollutants under sunlight. The regeneration studies demonstrated the possible reusability of the catalyst where only slight decrease (∼10 %) in the degradation efficiency was observed after five regenerations. The CMFE@ZnO NPs were also found to be promising antibacterial agents by inhibiting the growth of gram-positive and gram-negative bacterial strains. Interestingly, the NPs were found more active against gram-negative bacteria due to the thin cell membrane. Hence, the results show that these ZnO NPs produced through a biogenic route can be employed for the purification of polluted wastewater via photocatalytic degradation.

RETRACTED

## CRediT authorship contribution statement

**Abu Bakar Siddique:** Writing – review & editing, Writing – original draft, Methodology, Investigation. **Muhammad A. Shaheen:** Supervision, Project administration, Data curation, Conceptualization. **Azhar Abbas:** Writing – review & editing, Conceptualization. **Yasir Zaman:** Resources, Project administration. **Mohammed A. Bratty:** Investigation, Formal analysis. **Asim Najmi:** Writing – review & editing. **Ali Hanbashi:** Data curation. **Muhammad Mustaqeem:** Resources, Project administration. **Hassan A. Alhazmi:** Writing – review & editing, Resources, Funding acquisition. **Zia ur Rehman:** Investigation. **Khalid Zoghebi:** Resources, Formal analysis. **Hatem M.A. Amin:** Writing – review & editing, Visualization, Data curation, Conceptualization.

## Availability of data and materials

All evaluated data is available in the manuscript. Additional information/data can be provided upon reasonable request.

## Declaration of competing interest

The authors declare that they have no known competing financial interests or personal relationships that could have appeared to influence the work reported in this paper.
